The article "Drug-loaded erythrocytes: Modern approaches for advanced drug delivery for clinical use" was published in 2023. Journal: Heliyon.

# Drug-loaded erythrocytes: Modern approaches for advanced drug delivery for clinical use

**DOI:** 10.1016/j.heliyon.2023.e23451

**Published:** 2023-12-15

**Authors:** Kulzhan Berikkhanova, Erlan Taigulov, Zhanybek Bokebaev, Aidar Kusainov, Gulyash Tanysheva, Azamat Yedrissov, German Seredin, Tolkyn Baltabayeva, Zhaxybay Zhumadilov

**Affiliations:** a Center for Life Sciences, National Laboratory Astana, Nazarbayev University, Kabanbay Batyr 53, Astana, 010000, Kazakhstan; b University Medical Center, Nazarbayev University, Astana, 010000, Kazakhstan; c Astana Medical University, Astana, 010000, Kazakhstan; d Semey State Medical University, Semey, 071400, Kazakhstan; e Scientific-Production Center of Transfusiology, Astana, 010000, Kazakhstan; f Departament of Surgery, School of Medicine, Nazarbayev University, Kabanbay Batyr 53, Astana, 010000, Kazakhstan

**Keywords:** Targeted drug delivery, Red blood cells, Drug loading techniques, Hypo-osmotic drug encapsulation, Automatic production of drug-loaded RBCs

## Abstract

Scientific organizations worldwide are striving to create drug delivery systems that provide a high local concentration of a drug in pathological tissue without side effects on healthy organs in the body. Important physiological properties of red blood cells (RBCs), such as frequent renewal ability, good oxygen carrying ability, unique shape and membrane flexibility, allow them to be used as natural carriers of drugs in the body. Erythrocyte carriers derived from autologous blood are even more promising drug delivery systems due to their immunogenic compatibility, safety, natural uniqueness, simple preparation, biodegradability and convenience of use in clinical practice. This review is focused on the achievements in the clinical application of targeted drug delivery systems based on osmotic methods of loading RBCs, with an emphasis on advancements in their industrial production.

This article describes the basic methods used for encapsulating drugs into erythrocytes, key strategic approaches to the clinical use of drug-loaded erythrocytes obtained by hypotonic hemolysis. Moreover, clinical trials of erythrocyte carriers for the targeted delivery are discussed.

This article explores the recent advancements and engineering approaches employed in the encapsulation of erythrocytes through hypotonic hemolysis methods, as well as the most promising inventions in this field.

There is currently a shortage of reviews focused on the automation of drug loading into RBCs; therefore, our work fills this gap.

Finally, further prospects for the development of engineering and technological solutions for the automatic production of drug-loaded RBCs were studied.

The article "Drug-loaded erythrocytes: Modern approaches for advanced drug delivery for clinical use" was published in 2023. Journal: Heliyon.

Automated devices have the potential to provide the widespread production of RBC-encapsulated therapeutic drugs and optimize the process of targeted drug delivery in the body. Furthermore, they can expedite the widespread introduction of this innovative treatment method into clinical practice, thereby significantly expanding the effectiveness of treatment in both surgery and all areas of medicine.

## 1 Introduction

Scientific organizations worldwide are striving to create drug delivery systems that provide high local concentrations of a drug in targeted pathological tissue without affecting healthy organs in the body. Selective distribution of drugs by targeted delivery can induce the greatest therapeutic effect in the locally affected tissues and simultaneously reduce the overall toxicity of the drugs. To achieve this goal, different artificial synthetic drug delivery systems in medicine are currently being studied, for example, liposomes, dendrimers, micelles, fullerenes, and polymers [[1], [2], [3], [4], [5], [6], [7]]. However, most proposed artificial drug carriers have not yet received wide application due to considerable complexity in their preparation and complexation with drugs, restrictions on the drug dose to be bound, high cost, toxicity and immunogenic incompatibility.

The use of erythrocytes as drug carriers is a fundamental achievement in modern cellular bioengineering and can improve the treatment efficiency in many areas of medicine. Important physiological properties of red blood cells, such as frequent renewal ability, oxygen carrying ability, unique shape and membrane flexibility, allow them to be used as natural carriers of drugs in the body [8].

In recent years, there have been numerous review articles about promising innovative technologies based on engineered RBCs. Alongside the achievements in targeted drug delivery achieved through encapsulation within RBCs, a wide array of innovative technologies exists, including RBC membrane-camouflaged nanoparticles, RBC-derived extracellular vesicles and RBC-Hitchhiking. Most of these review articles summarize mainly preclinical studies conducted in vitro or using animal models [[8], [9], [10], [11], [12], [13], [14], [15]].

In this review, we aimed to highlight the achievements in the clinical application of targeted drug delivery systems based on osmotic methods of loading RBCs, with an emphasis on advancements in their industrial production. This article describes the fundamental techniques used to encapsulate drugs into erythrocytes obtained by osmotic methods, as well as the essential strategic approaches applied in clinical practice for targeted drug delivery using drug-loaded erythrocytes.

The article "Drug-loaded erythrocytes: Modern approaches for advanced drug delivery for clinical use" was published in 2023. Journal: Heliyon.

Moreover, clinical trials of erythrocyte carriers for the targeted delivery are discussed. This article explores the recent advancements and engineering approaches employed in the encapsulation of erythrocytes through osmotic techniques, as well as the most promising inventions in this field.

There is currently a shortage of reviews focused on the automation of drug loading into RBCs; therefore, our work fills this gap. More promising drug delivery systems are erythrocyte carriers derived from autologous blood due to their immunogenic compatibility, safety, natural uniqueness, simple preparation, biodegradability and convenience of use in clinical practice. The unique physiological properties of erythrocyte carriers are that they have the ability to improve the pharmacokinetics of drugs and provide biocompatibility and selective biodistribution of drugs in the human body, thereby increasing the effectiveness of therapy [16].

Automated devices have the potential to provide the widespread production of RBC-encapsulated therapeutic drugs and optimize the process of targeted drug delivery in the body. Furthermore, they can expedite the widespread introduction of this innovative treatment method into clinical practice, thereby significantly expanding the effectiveness of treatment in both surgery and all areas of medicine.

The main objective of this work is to explore the achievements in the clinical application of targeted drug delivery systems, with a specific focus on osmotic methods of loading RBCs. Moreover, the topical use of RBCs ghosts for targeted drug delivery is discussed as an emerging approach in clinical practice. Special attention is given to advancements in the industrial production of drug-loaded RBCs, as well as an investigation into potential future prospects.

## 2 Historical background

The first studies of adenosine triphosphate (ATP) loading in “erythrocyte ghosts” were reported by Gardos in 1954 [17]. Later works on drug loading of erythrocyte ghosts for the purpose of targeted delivery include the works by Marsden and Ostling (1959), Ihler et al. (1973) and Zimmerman (1975) [[18], [19], [20]]. Marsden and Ostling studied the penetration of dissolved dextran through the cell membrane after osmotic hemolysis and concluded that most of the absorbed dextran penetrated into the erythrocyte during hemolysis through a significant but temporary increase in membrane porosity, and the amount of residual hemoglobin in the cells was 49 % [18]. Ihler et al. demonstrated the possibility of incorporating two enzymes (β-glucosidase and β-galactosidase) into erythrocytes using cell hemolysis. They presumed that it may be possible to prepare enzyme-loaded cells capable of prolonged survival in the bloodstream, which could replace enzyme therapy [19]. Studies conducted by Zimmerman demonstrated the possibility of loading erythrocytes with the enzyme urease and indicated that these loaded ghost cells can release enzymes into the bloodstream during hemolysis [20]. The concept of “carrier erythrocytes” was first used in 1977 to characterize drug-loaded RBCs [21,22].

The article "Drug-loaded erythrocytes: Modern approaches for advanced drug delivery for clinical use" was published in 2023. Journal: Heliyon.

Unfortunately, shortly after these promising early studies exploring the concept of encapsulating pharmacological agents within isolated RBCs for the purpose of targeted drug delivery, the HIV pandemic, hepatitis, and other infections transmitted through blood products significantly impeded research in RBC-based drug delivery for several decades [13].

Nevertheless, several laboratories persistently developed biomedically valuable approaches for loading drugs into RBCs, advancing from in vitro proof of concept and studies in animal models to the current promising state [14,[23], [24], [25], [26], [27]].

Presently, alongside the achievements in targeted drug delivery achieved through encapsulation within RBCs, there exists a broad spectrum of innovative technologies. These encompass RBC membrane-camouflaged nanoparticles (RCNPs), red blood cell-derived extracellular vesicles (RBCEVs), and the concept of RBC-Hitchhiking [[8], [9], [10], [11], [12], [13], [14], [15]].

Currently, cargoes can be loaded into carrier RBCs using two main approaches: encapsulation of drugs within erythrocytes and surface loading of RBCs. The first approach involves encapsulating drugs within the inner space of RBCs. This can be achieved by inducing transient hypotonic swelling of cell membranes, followed by pore opening and subsequent resealing before reinfusion.

The second approach for loading drugs onto RBCs for delivery involves surface coupling of drugs or drug carriers. To foster objectivity and intellectual depth, we have opted to briefly explore the topic of surface loading of red blood cells in the next chapter.

## 3 Surface loading of RBCs - the second approach for loading drugs onto RBCs for delivery: mainly in the preclinical studies stage

The second approach for loading drugs onto RBCs for delivery involves surface coupling of drugs or drug carriers. There are various distinctive aspects that render surface loading a highly efficient alternative approach. Glassman et al. provided a concise overview of current technologies utilized for loading and coupling drugs with RBCs, emphasizing their impact on pharmacokinetics. Furthermore, this review provides a comprehensive description of changes in absorption, distribution, metabolism, and elimination, as well as highlighting the unique features of RBC pharmacokinetics [15].

The article "Drug-loaded erythrocytes: Modern approaches for advanced drug delivery for clinical use" was published in 2023. Journal: Heliyon.

In this study [28], the authors engineered single-chain antibody fragments (scFvs) from nonhuman primates targeting human RBCs. Then, these scFvs were fused with human thrombomodulin (hTM) to create a representative biotherapeutic cargo known as hTM-scFv. The engineered affinity ligands demonstrated a safe and effective method for coupling therapeutics to human RBCs. These results indicate that RBC-targeted scFv/TM exerts multifaceted cytoprotective effects and may find utility in systemic and focal inflammatory and ischemic disorders. The application of scFv/TM in mouse models to investigate systemic inflammation and ischemia-reperfusion injury has been examined [29]. The results indicated that RBC-targeted scFv/TM exerts multifaceted cytoprotective effects, suggesting potential utility in systemic and focal inflammatory and ischemic disorders. The authors propose these novel ligands as a potential solution to optimize the delivery of therapeutic drugs using human erythrocytes, with the aim of enhancing pharmacokinetics and antithrombotic effects.

Villa C.H. et al. [30] investigated the delivery of anti-inflammatory, antithrombotic, and antimicrobial agents bound to the surface of RBCs. They also explored the internal properties of erythrocyte membranes, immune-related aspects, potential surface targets, and methods for producing affinity ligands.

Murciano J.C. et al. [31] conjugated recombinant soluble urokinase plasminogen activator receptor (suPAR) to rat RBC, forming RBC/suPAR complex. The authors explored the coupling of plasminogen activators to rat RBCs and demonstrated an extension of their lifespan in the bloodstream, while also limiting side effects, making them suitable for short-term thromboprophylaxis.

In thise study [32] extensive research has been conducted to simulate the NPs detachment from RBCs hitchhiking under shear flow and flowing through microfluidic channels. This computational platform can be utilized as a predictive tool to estimate optimal parameters for NP-bound RBCs, enhancing targeting procedures within tissue microvasculature.

Ganguly K. et al. [33] studied the susceptibility of RBC/tPA to PA inhibitors including plasminogen activator inhibitor-1 (PAI-1) which can limit its function and shorten its efficacy. The results demonstrated that the RBC glycocalyx provides protection to RBC-coupled tPA against inhibition. Resistance to high levels of inhibitors in vivo contributes to the potential utility of RBC/tPA for thromboprophylaxis. The authors concluded, that coupling tissue-type plasminogen activator (tPA) to carrier RBCs extends its circulation in the bloodstream, making it suitable for thromboprophylaxis. Atukorale PU et al. introduced a system of amphiphilic gold nanoparticles (AuNPs) that, based on their core size and the hydrophobicity of their surface ligands, can become embedded within erythrocyte membranes. They have demonstrated that the embedding of amphiphilic AuNPs in erythrocyte membranes is influenced by membrane fluidity and the glycocalyx. Furthermore, the association of particles with RBC membranes is enhanced with higher temperatures up to physiological levels or the removal of the glycocalyx in general, especially sialic acids. These findings suggest that these amphiphilic AuNPs could serve as effective drug carriers, allowing for easy and swift embedding into erythrocyte membranes in vivo, without requiring prior ex vivo manipulation [34]. Glassman et al. highlighted the benefits of coupling drugs to the surface of RBCs. Coupling therapeutics to the RBC surface prevents membrane damage, which may occur during pore formation or transmembrane penetration required for internal encapsulation. This approach negates the necessity of releasing drugs encapsulated within red blood cells. Moreover, surface сoupling can be achieved in a single step, whether in vitro or in vivo [13].

The article "Drug-loaded erythrocytes: Modern approaches for advanced drug delivery for clinical use" was published in 2023. Journal: Heliyon.

Furthermore, surface loading facilitates RBC hitchhiking strategies. This involves coupling nanocarriers to the RBC surface, providing a range of benefits such as extending circulation time and transferring cargoes attached to RBCs to specific locations within the vasculature. Glassman P.M. et al. introduced a system of amphiphilic gold nanoparticles AuNPs that, based on their core size and the hydrophobicity of their surface ligands, can become embedded within erythrocyte membranes [35]. They have demonstrated that the embedding of amphiphilic AuNPs in erythrocyte membranes is influenced by membrane fluidity and the glycocalyx. Furthermore, the association of particles with RBC membranes is enhanced with higher temperatures up to physiological levels or the removal of the glycocalyx in general, especially sialic acids. These findings suggest that these amphiphilic AuNPs could serve as effective drug carriers, allowing for easy and swift embedding into erythrocyte membranes in vivo, without requiring prior ex vivo manipulation.

RBC-hitchhiking NPs exhibited remarkable brain localization levels, when utilizing intra-arterial catheters [36]. The technique of RBC hitchhiking has demonstrated successful application in various preclinical disease models, spanning from pulmonary embolism to cancer metastasis. Muzykantov et al. introduced the concept of RBC-hitchhiking (RH), in which nanocarriers (NCs) adsorbed onto RBCs transfer from RBCs to the first downstream organ upon intravascular injection. They demonstrated that optimized RH formulations can effectively and safely target NCs to specific organs through strategic placement of intravascular catheters in animal models. They proposed the use of RBC-hitchhiking for the treatment of acute respiratory distress syndrome, pulmonary embolism and acute ischemic stroke [37].

The article "Drug-loaded erythrocytes: Modern approaches for advanced drug delivery for clinical use" was published in 2023. Journal: Heliyon.

The Dual Targeted RBC Hitchhiking (DTRH) approach involves loading nanoparticles into circulating RBCs in vivo, expanding the range of vascular targets for drug delivery. Ferguson LT et al. proposed a novel strategy called DART - dual affinity to RBCs and target cells, in which nanocarriers are conjugated to two affinity ligands. One ligand binds to red blood cells, and the other binds to a specific target cell, such as pulmonary endothelial cells in this case [38]. The DART nanocarriers initially attach to red blood cells and then transfer to the endothelial cells of the target organs, facilitated as the bound red blood cells navigate through capillaries. The significant enhancement achieved by DART in both organ- and cell-type targeting holds potential for effectively localizing drugs in various medical applications. Utilizing cargoes with an affinity to RBCs allows for direct loading onto circulating RBCs, eliminating the need for isolating, loading, purifying, and re-infusing of the RBC drug delivery systems. This approach demonstrated promising results in animal studies, employing affinity fusion proteins that robustly bind to RBCs [30].

Numerous scientists are presently investigating the RBC-based drug delivery, and innovative strategies are coming to light, playing a significant role and driving groundbreaking discoveries. These approaches involve genetic molecular modifications of RBCs, immune system modulation through RBC-coupled antigens, and the vascular transportation of RBC-coupled nanocarriers, known as RBC hitchhiking [14,31,[39], [40], [41], [42], [43], [44], [45]].

Measuring the concentration of injected substances within the body poses a significant challenge. Due to regulatory constraints and related issues, this situation contributes to the limited research focused on quantitatively analyzing blood pharmacokinetics, biodistribution, clearance, and the prolonged circulation time of carrier RBCs and their cargo. The available semi-quantitative studies generally indicate that drugs loaded into RBCs circulate for extended periods and display different biodistribution compared to their free counterparts [32]. However, conducting more comprehensive studies to quantitatively assess the influence of RBC modification on its pharmacokinetics and biodistribution is essential. The encapsulation of drugs within RBCs usually leads to enhanced pharmacokinetics (PK) compared to free drugs, ultimately improving effectiveness in animal models and patient outcomes. The authors [15] have provided an in-depth explanation of crucial ADME (absorption, distribution, metabolism, elimination) changes expected for drugs associated with RBCs and have highlighted specific aspects of RBC pharmacokinetics. The authors [35] outlined methods for initial in vitro testing of the biocompatibility of modified and drug-loaded RBCs. These assessments included evaluating aggregation, complement fixation, hemolysis, resistance to mechanical stress, translocation of PS to the RBC surface, and the level of CD47.

The article "Drug-loaded erythrocytes: Modern approaches for advanced drug delivery for clinical use" was published in 2023. Journal: Heliyon.

The established method to enhance pharmacokinetics involves coating nanoparticles with polymers, particularly polyethylene glycol (PEGylation), a technique widely utilized in various clinically approved products. In vitro experiments examined antibody-mediated binding of liposomes to erythrocytes to determine a suitable loading dose that wouldn't harm the carrier cells. When erythrocyte-targeting liposomes were administered to mice, there was an approximate twofold increase in the area under the blood concentration-time curve compared to PEGylated liposomes. RBC ligands targeting glycophorin A (GPA) and band 3 can cause undesired changes in RBC properties, including deformability modifications, exposure of phosphatidylserine (PS), and reactive oxygen species (ROS) generation. Antibodies against GPA and band 3 usually reduce membrane deformability. The effects on the membrane vary, even among epitopes within the same target protein. Surface proteins may have crucial intrinsic functions that ligand binding could disrupt, such as GPA's interaction with neutrophils for quiescence or ion transport by band 3. Thorough investigation of adverse effects is essential to identify optimal RBC targets and ensure no adverse impact on RBC physiology. The ideal target should be specific to erythroid cells, adequately abundant for therapeutic intent, widely distributed among human populations, and not compromise RBC biocompatibility [28,38,46].

Studies of the immunogenicity of erythrocyte carriers have been carried out. Luk B.T. et al. [47] explored a nanoparticle platform coated with a cell membrane, investigating its potential as a drug delivery vehicle for treating a murine model of lymphoma. They examined the feasibility of employing a biomembrane-coated approach to design nanocarriers that are functional, safe, and immunocompatible for delivering cancer drugs. The study demonstrated that this approach efficiently delivered a model chemotherapeutic agent, doxorubicin, to solid tumor sites, significantly augmenting the suppression of tumor growth compared to conventional free drug treatment. Hanley T.M. et al. have developed erythrocyte-derived particles incorporating indocyanine green activated by near-infrared (NIR) light for applications in phototheranostics. A critical concern regarding the clinical implementation of these particles involves their potential immunogenic effects. The researchers assessed the acute phase of the innate immune response triggered by these particles in healthy mice after tail vein injection. This assessment involved measuring specific cytokine levels in the blood serum, liver, and spleen following euthanasia. Cytokine response to nanosized particles exhibited statistically significant elevations in IL-6 in the liver and spleen, TNF-α in blood serum, the liver, and the spleen, and MCP-1 in the liver and spleen as compared to PBS-induced levels. The results revealed that the functionalization of these nanosized particles led to a reduction in IL-6 and MCP-1 levels in the blood serum, liver, and spleen, as well as a decrease in TNF-α levels in the blood serum [48]. Sun L. et al. packaged Prussian blue (PB) nanoparticles within Chlorin e6 (Ce6)-imbedded erythrocyte membrane vesicles, named as PB@RBC/Ce6 NPs. This innovative approach allowed them to leverage both the biological properties of natural erythrocyte membranes and the distinctive physicochemical characteristics of synthetic nanoagents. In comparison to bare PB NPs or free Ce6, PB@RBC/Ce6 NPs demonstrated significantly heightened cellular uptake and accumulation in tumoral tissues. Moreover, they exhibited a noticeable ability to induce necrosis and late apoptosis of tumor cells in vitro, and showed a synergistic therapeutic effect against an orthotopic tumor model in vivo [49].

The article "Drug-loaded erythrocytes: Modern approaches for advanced drug delivery for clinical use" was published in 2023. Journal: Heliyon.

There are also alternative approaches to encapsulating drugs in erythrocyte carriers, involving the use of peptides that penetrate the cell in association with the encapsulated compound [23,[49], [50], [51]]. Sabatino et al. investigated using RBCs as a carrier to target bisphosphonates to macrophages for elimination, both in vitro and in vivo. RBCs loaded with bisphosphonate Zoledronate were found to be effective for targeted delivery to macrophages in both settings [51].

Lu et al. [52] emphasized the importance of membrane mechanical properties as a key criterion in the design and development of RBC-based delivery systems. To achieve this goal, they used optical methods combined with image analysis and mechanical modeling. Lu et al. provided quantitative information on the morphological characteristics, hemoglobin content, and mechanical properties of the membranes of a red blood cell-based delivery system incorporating the FDA-approved near-infrared material, indocyanine green. Their findings indicated notable alterations in material properties in these particles. Consequently, the membrane of these particles exhibited reduced deformability and heightened resistance to flow. The authors attributed these changes to impaired membrane–cytoskeleton attachment in the particles.

Coating nanoparticles with cell membranes is a strategy used in nanomedicine to improve the nanoparticles' biocompatibility and circulation time in the bloodstream. Red blood cell membranes (RBCM) have been used for external coating of synthetic NPs containing therapeutic agents to produce RBC membrane-camouflaged nanoparticles (RCNPs).

RCNPs represent an exceptional nanocarrier platform that synergizes the immunomodulatory attributes of natural cellular components with the cargo-carrying capabilities of polymeric nanoparticles. RCNPs have been developed to treat various diseases with promising preclinical results.

Extracellular vesicles (RBCEVs), derived from red blood cells and naturally released by them, serve as carriers for drug delivery. These RBCEVs play a pivotal role in intercellular communication, maintaining homeostasis, and modulating the immune system under both physiological and pathological conditions [[13], [14], [15]]. Due to these essential functions, extracellular vesicles originating from red blood cells offer a promising strategy for the treatment of various pathologies. Developing reliable methods for the more efficient isolation of a substantial quantity of extracellular vesicles, obtained from erythrocytes, is crucial for their clinical application.

Despite the significant advances made by RCMP and RBCEV-based platforms in tackling pivotal challenges within the field of nanodrug delivery, these platforms still face with various issues. One such challenge belongs to the incongruity between positively charged NP surfaces and the RBCM coating, which constrains the applicability of RCNP systems [8,9,[13], [14], [15]].

The concept of RBC hitchhiking is based on nanocarriers' ability to non-covalently adhere to the surface of RBCs and subsequently detach from the RBCs within small blood vessels, thereby facilitating their delivery to the to the target site. The RBC-hitchhiking strategy offers a range of benefits, including prolonging circulation time and transporting RBC-coupled cargoes to specific sites within the vasculature. However, RBC hitchhiking technology still requires further investigation before transition from research circumstances to industrial and clinical applications [[13], [14], [15]].

The article "Drug-loaded erythrocytes: Modern approaches for advanced drug delivery for clinical use" was published in 2023. Journal: Heliyon.

Thus, the achievements obtained with RCNPs, RBCEVs and RBC hitchhiking technologies have incomplete substantiation from safety studies conducted in animal models, and there is an insufficient amount of information available concerning potential complications associated with the combination of biological and synthetic materials.

Therefore, there is a pressing need for the further development of the most promising RBC-based drug delivery systems. The emphasis should be on optimizing technologies such as RCNPs, RBCEVs, and RBC hitchhiking, as well as large-scale production processes to utilize RBCs effectively as carriers for nanoparticles [14,15]. We would like to emphasize the importance of taking into account the physicochemical and mechanical properties of the membrane when engineering erythrocyte-derived carriers. This consideration is especially crucial in the context of ensuring the safe and effective clinical translation of erythrocyte-derived platforms. It is crucial to highlight that studies on the surface loading of RBCs are currently in the preclinical stage of investigation, conducted in vitro or using animal models.

## 4 Basic methods for encapsulating drugs into red blood cells

The feasibility of targeted delivery of various drugs by encapsulation in RBCs has been proven by numerous experimental and clinical studies [1,[53], [54], [55], [56]]. Many methods for creating drug delivery systems based on RBCs have been published. Currently, there are several basic methods for encapsulating drugs into red blood cells, such as electroporation, pharmacologically induced endocytosis, the osmotic pulse method, and hypotonic hemolysis [[57], [58], [59], [60]].

The essence of the electroporation method is that cells placed in an isotonic solution are exposed to a high-voltage electric field. Under the influence of an electric current, the permeability of the cell membrane increases, ions are exchanged through the membrane, and the drug molecules enter the erythrocytes from the extracellular fluid [[61], [62], [63]].

Pharmacologically induced endocytosis is based on the ability of the plasma membrane to absorb extracellular substances into the cell through the small vesicles formed by the invagination of the plasma membrane [[64], [65], [66]].

The necessity of employing specific preparations to load drugs into erythrocytes through endocytosis seems to emphasize the absence of a natural endocytosis pathway in erythrocytes. Endocytosis in erythrocytes appears to occur exclusively through « drug-induced endovesiculation » or « pharmacologically induced endocytosis». Furthermore, recent publications have indicated that drug molecules can permeate RBCs through endocytosis in the presence of specific chemical compounds. For instance, primaquine, vinblastine, chlorpromazine, hydrocortisone or tetracaine have been reported to induce this process [[58], [59], [60],^67^,^68^].

The article "Drug-loaded erythrocytes: Modern approaches for advanced drug delivery for clinical use" was published in 2023. Journal: Heliyon.

Walter Oberwagner et al. investigated drug-induced endovesiculation of freshly prepared human erythrocytes [69]. Cationic amphiphilic drugs such as chlorpromazine are recognized to induce a cup-like cell shape and vesicle formation within the cell. The authors examined various conditions influencing endovesiculation induced by chlorpromazine. They observed that inhibitors of membrane fluctuations, such as ATP depletion, vanadate, or fluoride, were effective in inhibiting endovesiculation. Conversely, activation of PKC, known to reduce cytoskeleton association and increase membrane fluctuations, enhanced endovesicle formation. This suggests that the formation of endovesicles and membrane fluctuations are regulated by similar cytoskeleton-driven membrane properties.

Ginn et al. discovered that endocytosis may be induced in mature erythrocytes by drugs of a specific chemical structure. Molecules intercalate passively into the inner membrane of the phospholipid bilayer of the erythrocytes. This process ends with the formation of vacuoles (containing the drug) within the intraerythrocytic compartment. The performance of the process is dependent on drug concentration, pH (7.9–8.1), and temperature (37 °C). However, the method is only suitable for the entrapment of cations or anions, which have both hydrophobic and hydrophilic groups. This limitation combined with an evident lack of process reproducibility makes it incompatible with an industrial development [60,70].

However, in recent decades, as understanding of the complex molecular mechanisms of endocytosis and the resilient mechanical properties of the erythrocyte membrane framework induced by the spectrin-actin network deepened, reports have emerged suggesting that erythrocytes were incapable of undergoing endocytosis. This viewpoint is attributed to the absence of a molecular mechanism in erythrocytes for the formation and internalization of endocytic vesicles [71,72].

The osmotic pulse method was developed by Franco et al., in 1987. In this method, an osmotic impulse causes temporary openings in a cell membrane through which a drug can penetrate into RBCs. This technique is based on the rapid diffusion of dimethyl sulfoxide (DMSO) through the cell membrane and includes the following steps: incubation of an erythrocyte suspension in DMSO solution, isotonic dilution of the erythrocytes with the drug solution, incubation of the suspension after dilution and, finally, restoration of the membrane and return of the cells to their initial state [73,74]. Al-Essa et al. [75] conducted a study focusing on the swift loading of RBCs using fluorescent antibodies and a nuclear staining dye, exploring their potential bioanalytical applications. The objective of this study was to load various antibodies (Abs) and a fluorescent dye onto the RBCs. The DMSO conservation step proved sufficient in rendering the RBCs reactive for the insertion of specific Abs and fluorescent dyes. This step led to a substantial increase in fluorescence signals, suggesting significantly enhanced RBC loading capacity.

The article "Drug-loaded erythrocytes: Modern approaches for advanced drug delivery for clinical use" was published in 2023. Journal: Heliyon.

The authors [76] utilized two- and three-component synthetic membranes (liposomes) as well as the plasma membrane of human erythrocytes to explore the impact of adding DMSO to the membrane-solvating environment. The experimental findings indicate that DMSO is likely to exert varying effects on heterogeneous biological membranes, contingent upon their local composition and structure. Moreover, DMSO could potentially influence membrane-associated biological functions. The authors demonstrated that DMSO modifies the elasticity of the RBC membrane and increases membrane permeability to ATP, even at relatively low concentrations of DMSO. Plenge-Tellechea F. et al. [77] assessed the impact of chlorpromazine (CPZ) and DMSO on the hydrolytic activity of plasma membrane Ca2+-ATPase (PMCA). In the absence of CPZ, DMSO causes a gradual reduction in activity. However, in the presence of CPZ, the activity profile against DMSO shifts, resulting in a recovery of activity. This suggests a potential partitioning of CPZ influenced by the solvent. The authors [78] utilized thermal dielectroscopy to investigate the effects of formamide, N-methylformamide, N,N-dimethylformamide and dimethyl sulfoxide on the segmental mobility and binding of the spectrin-based skeleton to the lipid membrane of human erythrocytes. The DMSO method yields highly loaded RBCs, but only a small fraction of cells (approximately 9%–25 %) are affected. To isolate this cell fraction, researchers have employed a Percoll separation. However, this method proves to be time-consuming and expensive, making it primarily suitable for only laboratory-scale applications [60]. DMSO finds extensive use in various biological and biotechnological applications, primarily due to its impact on the cell plasma membrane, including RBCs. However, the precise molecular mechanisms underlying this action are still not fully understood.

The inclusion of chemotherapeutic drugs in RBCs by hypotonic hemolysis is generally recognized as a clinically proven and widespread technique [57]. Notably, there is a fairly large range of modifications of the method of hypotonic hemolysis. The four most common methods are hypotonic preswelling, hypotonic dialysis, hypotonic dilution, and hypoosmotic hemolysis (Fig. 1).

The article "Drug-loaded erythrocytes: Modern approaches for advanced drug delivery for clinical use" was published in 2023. Journal: Heliyon.

**Fig. 1:** Basic methods for incorporating drugs into red blood cells. Flowchart of the main methods of including drugs in red blood cells with a focus on the hypotonic hemolysis method. (For interpretation of the references to colour in this figure legend, the reader is referred to the Web version of this article.)

The principle of this method is cell lysis after cell swelling and reaching a critical volume and pressure (Fig. 2). Multiple holes with diameters of 20–50 nm appear on the cell membrane, allowing various drugs in the lysing solution to enter the cell. It was also found that on average, 1/3 of the total cell volume can be replaced with a lysing solution. Thus, red blood cells can include not only corticosteroids and enzymes but also proteins, lipids, DNA, cytokines, antibiotics, anticancer drugs, etc. After the concentration of the lysing solution is restored to isotonic, the integrity of the membrane is restored [[57], [58], [59]].

**Fig. 2:** The procedure of RBC drug loading using hypotonic hemolysis. Schematic of the preparation process of RBC drug loading using hypotonic hemolysis. 1-isotonic solution; 2-erythrocyte; 3-swelling of erythrocytes; 4-hypotonic solution; 5- substance for encapsulation; 6-RBCs have reached critical volume and pressure; 7-pharmacocytes - drug loaded RBCs; 8-isotonic solution.

Most medicines and diagnostic drugs are encapsulated into red blood cells through the abovementioned mechanisms of hypotonic hemolysis. For example, the hypotonic preswelling method was demonstrated by Rechsteiner M.C., who modified the techniques of Tajerzadeh H. and Hamidi M [79,80]. The hypotonic preswelling method was also commonly used by Magnani M. et al. as a delivery technique for dexamethasone encapsulated into erythrocytes [[81], [82], [83], [84], [85], [86], [87], [88], [89]]. Godfrin Y. et al. applied the hypotonic dialysis technique for encapsulating drugs into red blood cells [90,91]. The hypotonic dilution method was used by Ihler G. and Updike S. J. et al. to investigate the encapsulation of enzymes, lipids, asparaginase, etc., into red blood cells [57,91]. Zhumadilov Zh. et al. used the technique of hypoosmotic hemolysis to study the possibility of using targeted transport of antibiotics in autologous erythrocyte ghosts in the treatment of acute cholecystitis patients older than sixty years. The high clinical efficiency of the hypoosmotic hemolysis technique was proven, but the difficulty of introducing the technique into wide clinical practice was also emphasized [92,93].

The article "Drug-loaded erythrocytes: Modern approaches for advanced drug delivery for clinical use" was published in 2023. Journal: Heliyon.

It's crucial to emphasize that within the body, macrophages identify any mechanical, biophysical, and biochemical alterations in the properties of erythrocyte membranes that occurred during their loading as indicators of apoptotic or aging erythrocytes. The RBC membrane acquires internal structural support from its cytoskeleton, specifically the hexagonal actin–spectrin lattice that acts as its foundation. This lattice interconnects with anchoring and membrane proteins, such as glycophorin A and band 3 protein, which are among the most abundant integral glycoproteins within the extensive array of proteins found in the RBC plasma membrane [30].

The distinct membrane properties of RBCs stem from the interaction between the plasma membrane envelope and the cytoskeleton [94]. The plasma membrane is constructed from a lipid bilayer with transmembrane proteins embedded within, forming multi-protein complexes. This bilayer is composed of an equal balance of cholesterol and phospholipids. To maintain structural integrity, the bilayer is interconnected with the membrane skeleton through two macroprotein complexes: the ankyrin complex and the junctional complex, also referred to as the 4.1R complex. The RBC skeleton constitutes a protein meshwork, wherein the most important components include spectrin, actin, actin-associated proteins, protein 4.1R, and ankyrin. The normal RBCs possess highly flexible biomechanical properties. Their characteristic discoid biconcave shape grants them a considerable surface-to-volume ratio (∼1.5), allowing for notable and reversible deformations essential for navigating through narrow capillaries repeatedly.

This distinctive shape, offering about 40 % more surface area compared to a sphere of the same volume, in conjunction with the specific structural organization of regular RBCs, serves as the primary factor determining their mechanical attributes. The robust adherence between the membrane bilayer and the cytoskeleton plays a crucial role in upholding the membrane surface area. This adherence is established through connections between the intracellular domains of membrane proteins and the spectrin-based cytoskeleton network.

Key connections are facilitated by membrane proteins such as Band and RhAG, linked to the spectrin network via Ankyrin, and glycophorin C, XK, Rh, and Duffy, which establish the linkage via protein 4.1R. Additionally, the binding of PS to cytoskeletal proteins and the spectrin network significantly contributes to the mechanical stability and deformability of regular RBCs.

The article "Drug-loaded erythrocytes: Modern approaches for advanced drug delivery for clinical use" was published in 2023. Journal: Heliyon.

Within the lipid bilayer of RBCs, four major phospholipids exhibit an asymmetric distribution: phosphatidylcholine and sphingomyelin are predominantly located in the outer leaflet, whereas phosphatidylethanolamine and anionic phosphatidylserine (PS) are situated in the inner leaflet.

The placement of PS in the inner layer of regular RBCs is facilitated by an ATP-dependent aminophospholipid translocase (flippase) which swiftly moves PS from the outer to the inner layer. This function relies on the intracellular concentration of Ca+2 and is likely associated with a P-type Mg2+-ATPase, with ATP11C identified as a flippase [95,96]. Jia W et al. conducted an extensive investigation into the circulation dynamics of micron and nano-sized erythrocyte-derived carriers within the vasculature of mice using real-time near-infrared fluorescence imaging. They meticulously examined the physicochemical characteristics of the membrane and the role of phosphatidylserine in the clearance of these particles [95]. Tang et al. demonstrated that membrane cholesterol enrichment of Red Blood Cell-Derived Microparticles can lead to their long-term circulation [96]. The flipping of phosphatidylserine from the inner to the outer membrane leaflet normally occurs during the manufacture of such particles. PS externalization serves as a signal for the phagocytic removal of the particles from circulation. The authors demonstrated that membrane cholesterol enrichment can alleviate the outward presentation of PS on microparticles derived from RBCs. In vitro findings indicated that murine macrophages exhibit a decreased uptake rate for cholesterol-enriched particles, resulting in reduced ingestion compared to RBC-derived particles without cholesterol enrichment. These results indicate that membrane cholesterol enrichment is an effective approach for reducing PS externalization on the surface of RBC-derived particles and prolonging their presence in circulation. Lee CH et al. conducted a comprehensive analysis of proteomes within erythrocyte ghosts of both micro and nanoscale, loaded with indocyanine green. They compared these proteomes to that of intact RBCs using techniques such as sodium dodecyl sulfate-polyacrylamide gel electrophoresis (SDS-PAGE) and quantitative tandem mass tag mass spectrometry, in conjunction with bioinformatics analysis [97]. In their study, a total of 884 proteins were identified in each set of RBCs, micro-sized particles, and nanosized particles. Notably, 8 proteins exhibited significantly different relative abundances when comparing micro-sized particles to RBCs, and 45 proteins showed this difference in the case of nanosized particles versus RBCs. The authors observed more pronounced variations in the relative abundances of certain mechano-modulatory proteins, such as band 3 and protein 4.2, and immunomodulatory proteins like CD44, CD47, and CD55 in nanosized particles compared to RBCs. These findings underscore the considerable influence of the methods used in the manufacture of RBC-based systems on their proteomes.

The article "Drug-loaded erythrocytes: Modern approaches for advanced drug delivery for clinical use" was published in 2023. Journal: Heliyon.

The authors [98] developed high-throughput in vitro assays to evaluate the vulnerability of NPs loaded RBCs to osmotic stress, mechanical, oxidative stress, and complement insults. The results indicate that mouse RBCs are more susceptible to these damaging factors compared to human RBCs. Loading RBCs with NPs at a 1:50 ratio showed no significant impact. However, increasing the NP load by 10–50 times worsened RBC damage from mechanical, osmotic, and oxidative stress. Additionally, excessive NP loading caused RBCs to aggregate in the buffer.

This study [99] delves into the challenges related to the activation of the alternative complement pathway by modified RBCs and explores strategies aimed at overcoming this issue. The authors highlighted the importance of CD47 and complement inhibitors such as DAF, CD59, and CR1 in preserving the biocompatibility of native RBCs. They investigated the mechanisms behind biotin-avidin-induced lytic susceptibility, specifically analyzing the impact of biotinylation and avidin cross-linking on key E complement regulatory molecules, decay accelerating factor (DAF), and CD59. During the loading of erythrocytes, the membrane experiences an osmotic effect, influencing the integrity, flexibility, and mechanical robustness of both the erythrocyte membrane and cytoskeleton. Exposure of phosphatidyl serine (PS) increases [100]. These alterations result in complement fixation and its activation, deformation of RBCs, and heightened sensitivity to various stresses, including mechanical, oxidative, and immunological stresses. The impact of PS on erythrocytes has also been linked to the activation of coagulation. All these unintended consequences of erythrocyte loading can potentially result in serious side effects. It is crucial to highlight that the relocation of PS to the outer layer is a distinctive feature of RBCs undergoing apoptosis, labelling them for phagocytosis by macrophages that possess PS receptors recognizing externally exposed PS on apoptotic RBCs. Additionally, the exposure of PS on the cell surface is linked to the elimination of senescent normal RBCs by macrophages in the spleen [95,96].

We would like to emphasize that the alterations in the mechanical, physical, and biochemical properties of erythrocyte membranes during their loading can vary depending on the loading technique and the specific chemicals employed during incubation.

The article "Drug-loaded erythrocytes: Modern approaches for advanced drug delivery for clinical use" was published in 2023. Journal: Heliyon.

## 5 The main strategic approaches used in clinical applications of erythrocyte-based cellular transport systems

Several strategies for the clinical application of drug delivery procedures based on osmotic loading of erythrocytes have been described in the literature [16,54,56].

Namely, the following main strategic approaches of RBC-based cellular transport systems are in use for clinical application:

1. targeted drug delivery to the systemic circulation.
2. targeted drug delivery to the reticuloendothelial system (RES).
3. topical use of RBC ghosts for targeted drug delivery.

In the first approach, the RBC ghosts are used as circulating bioreactors and for the gradual release of the encapsulated drug. Enzyme-encapsulated erythrocytes are called RBC bioreactors [60,74]. Encapsulation of enzymes in erythrocytes prevents early inactivation of these enzymes by preventing direct contact with plasma proteases. Exogenous toxins or pathological metabolites in the blood penetrate erythrocyte carriers, where they react with the encapsulated enzyme. RBC bioreactors are used in congenital enzyme deficiency in enzyme replacement therapy and in the removal of external toxins. In this case, erythrocyte carriers act as a reservoir for the drug and allow a gradual release of the encapsulated drug [60]. The gradual release of the encapsulated drug creates a constant presence of a certain stable concentration of the drug in the blood plasma and increases the duration of circulation of the drug in the bloodstream, thereby enhancing its therapeutic effect.

This approach prevents a simultaneous increase in the peak concentration of the free drug in plasma during intravenous administration of the drug, which reduces side effects and the toxicity of the drug, as well as the frequency of injections and the daily dose [93].

Erythrocyte carriers prevent the binding of the drug to plasma proteins, which preserves the activity of the drug and prevents immunological conflicts.

The second approach is based on the monocyte–macrophage system of internal organs (spleen, liver), where, according to physiology, aging or damaged erythrocytes undergo phagocytosis and are digested, which is a form of natural elimination. At the same time, the maximum concentration of the drug loaded into carrier RBCs is released in the target region of the reticuloendothelial system. Carrier erythrocytes loaded with the drug are recognized by macrophages as damaged cells; therefore, they are captured and digested. Upon phagocytosis of pharmacocytes, the drug concentration reaches a maximum for a longer time in the target region [60,93].

The article "Drug-loaded erythrocytes: Modern approaches for advanced drug delivery for clinical use" was published in 2023. Journal: Heliyon.

The topical application of drugs deposited in RBC carriers results in modification of the pharmacokinetics of drugs [[101], [102], [103]]. Local introduction of RBC-encapsulated antibiotics in a pathological inflammatory region allows the creation of a high local and prolonged concentration of the drug compared to the traditional use of a free drug. This approach is justified by the physiological nature of the inflammatory process. Purulent tissues have a more intensive blood supply and a high number of macrophages.

Autologous erythrocyte carriers containing an antibiotic are selectively captured by cells of the macrophage system. The release of the active drug from erythrocyte carriers occurs mainly during phagocytosis. Directly in the purulent-inflammatory region, phagocytosis of many pharmacocytes occurs with the release of a high concentration of the encapsulated drug [[101], [102], [103]].

Thus, modification of the pharmacokinetics of drugs deposited in cell carriers makes it possible to create a highly stable concentration of drugs in tissues where the inflammatory process is maximally manifested [92,102,103].

The main strategic approaches of targeted drug delivery based on osmotic loading of erythrocytes used in clinical practice are shown in Fig. 3.

**Fig. 3:** The main approaches to the clinical application of erythrocyte-based drug delivery. Schematic diagram of key strategic approaches for targeted drug delivery based on the osmotic loading of erythrocytes used in clinical practice.

## 6 Clinical use of erythrocyte carriers for the delivery of therapeutic agents

Recently, the use of RBCs for drug delivery has been increasingly expanding toward clinical use both in therapy and in the diagnosis of many diseases [16,54,56,88].

The unique physiological advantages of erythrocytes, especially autologous erythrocytes, in targeted drug delivery open up wide opportunities for clinical application and standardization of the construction of these drug delivery systems.

Cellular delivery systems based on autologous erythrocytes have been introduced into clinical practice in many countries. An example is the official recognition and decision of the European Medical Agency (EMA) to register the use of erythrocyte-mediated delivery of dexamethasone 21-phosphate in steroid-dependent ulcerative colitis as an orphan technology [81].

Several phase I/II clinical trials have been conducted that demonstrate the clinical efficacy of using Dexa 21-P-loaded RBCs in the treatment of patients with chronic obstructive pulmonary disorder (COPD), cystic fibrosis, Crohn's disease, ulcerative colitis and ataxia-telangiectasia [[81], [82], [83], [84], [85]]. Magnani M. et al. emphasized carrier erythrocytes, highlighting them as a highly promising drug-delivery systems, naturally designed as carriers, and their versatility in the realm of biologics for treating diverse pathological conditions. Utilizing erythrocytes as carriers for different drugs helps minimize toxicity, reducing the risk of side effects and pathological immune responses against encapsulated agents. This approach enhances drug efficacy, ultimately improving patient compliance [86].

The article "Drug-loaded erythrocytes: Modern approaches for advanced drug delivery for clinical use" was published in 2023. Journal: Heliyon.

Magnani M. anticipates that in the coming years, clinical applications will unquestionably receive approval from regulatory bodies and become accessible to the entire patient community, extending beyond those currently involved in various ongoing clinical trials [87].

The results of one study [89] demonstrated that the derivative corticosteroid dexamethasone 21-phosphate (Dexa 21-P) was detected in the bloodstream of volunteers within a month after a single injection of the drug loaded into autologous RBCs. Studies by Domenech C. et al. [90] revealed the circulation of asparaginase loaded into red blood cells for 30 days in the blood of patients.

There are numerous articles aimed at specific areas of application of erythrocyte delivery systems. The clinical use of erythrocyte carriers for the delivery of therapeutic agents in oncological, neurological, cardiovascular, metabolic, infectious and other diseases, as well as for imaging and diagnostics, are considered in the reports [67,104,105]. Koleva L. et al. concluded that carrier erythrocytes would be widely used, especially in enzyme replacement and antitumor therapy, soon [67]. However, the authors noted the complexity of the industrial production of drug-loaded erythrocytes, since RBC-based targeted drug delivery is a type of personalized medicine and requires a special approach. Mao Y. et al. considered recent advances in clinical trials of erythrocyte delivery systems and satisfactory results in cancer treatment [104]. The authors identified four main areas of application of erythrocyte carriers in cancer therapy that showed good results: enzyme-based cancer therapy, delivery of medicines, combination with nanoparticles and different anticancer agents. Drug delivery systems are attracting increasing interest due to their ability to increase the effectiveness of chemotherapeutic drugs, such as antitumor cytostatic drugs. Targeted delivery of a chemotherapeutic drug creates high concentrations of the drug in the foci of a cancerous tumor, enhances the clinical efficacy and bioavailability of anticancer drugs, and can also help reduce overall toxicity due to selective drug distribution in the body. l-Asparaginase encapsulated in erythrocytes has been used in clinical studies of acute lymphoblastic leukemia in children and adults for the treatment of asparagine-deficient malignancies [105]. The clinical use of enzyme-loaded RBCs as delivery systems has resulted in improved pharmacodynamics of l-asparaginase and effective protection against proteolytic enzymes circulating in the blood.

The article "Drug-loaded erythrocytes: Modern approaches for advanced drug delivery for clinical use" was published in 2023. Journal: Heliyon.

Javed S. et al. [106] summarized recent advances in the delivery of nanoerythrosome-based anticancer drugs for the therapy and diagnosis of various tumors. Various therapeutic approaches have been considered for erythrocyte-based enzymatic therapy for detoxification of exogenous chemicals, thrombolytic therapy, enzyme therapy and antitumor therapy [107].

Clinical applications of erythrocyte-mediated delivery and cell therapy in terms of transfusion-based medicines and blood component preparation procedures have been discussed in previous works [108,109]. The authors noted the benefits and preferences of developing optimal loading protocols, using sealed sterile procedures to avoid contamination and limiting the use of drug-loaded RBCs within 24 h.

An effective method for the erythrocyte-based targeted delivery of various antibiotics, hepatoprotectors, cytokines, etc., has been developed for the treatment of cholecystitis, peritonitis, purulent wounds and septic conditions [92,93,101,[110], [111], [112]]. The drug-loaded RBCs obtained through the method of hypo-osmotic hemolysis are conventionally referred to as “pharmacocytes.” The microphotographs presented in Fig. 4 show the morphological alterations of erythrocytes during drug encapsulation using the hypo-osmotic hemolysis method, as captured using scanning electron microscopy (Fig. 4A and B,C).

**Fig. 4:** Morphological alterations of erythrocytes during drug encapsulation using the hypo-osmotic hemolysis method. Scanning electron microscope images: A - Intact erythrocytes after washing three times. B - erythrocytes after addition of distilled water. C - Drug-loaded RBCs after “resealing”.

Electron microscopic studies have revealed that when RBCs are exposed to a hypotonic solution, their shape transitions from biconcave (Fig. 4A) to spherical (Fig. 4B). By reducing the tonicity of the solution through dilution with distilled water, the erythrocyte membrane swells and forms adequately large pores, enabling the exchange of cell contents with the external environment. Conversely, an increase in the tonicity of the incubation solution leads to the restoration of the erythrocyte membrane, returning it to its original biconcave shape, that apparently shows the “resealing” of the membrane (Fig. 4C).

The article "Drug-loaded erythrocytes: Modern approaches for advanced drug delivery for clinical use" was published in 2023. Journal: Heliyon.

Zhumadilov Zh. and Makarenkova R. conducted preclinical research and proved the feasibility of the effective encapsulation of antibiotics in RBC ghosts by hypo-osmotic hemolysis [92]. According to the research data, kanamycin and gentamicin showed the best loading into RBCs [92]. Zhumadilov Z. and Taigulov E. used targeted delivery of antibiotics in autologous erythrocyte ghosts for the treatment of acute cholecystitis patients older than 60 years, and high clinical efficacy was observed [101,110]. The targeted delivery of antibiotics loaded in erythrocyte ghosts has been used in the treatment of patients with purulent inflammatory diseases of the hepatobiliary system and septic conditions. The high efficiency of this method in comparison with the traditional intravenous administration of the same dose of free drugs has been proven [110,111]. An original method for the treatment of patients with anal abscesses has been developed and introduced into clinical practice [101,112]. Standard surgical treatment of abscess cavities was performed by opening, sanitizing, and excising necrotic tissues. Then, the edges and bottom of the wound were treated with erythrocyte pharmacocytes containing a single dose of an antibiotic. Primary sutures were applied to the wound. This method to treat anal abscesses accelerated the wound healing process, created conditions for the primary healing of a purulent wound, decreased the duration of treatment and reduced the frequency of relapses. The method had good functional and cosmetic effects [101,112].

A new method for the local treatment of purulent wounds by topical application of autologous pharmacocytes containing antibiotics and cytokines has been developed for use in preclinical studies. The pharmacokinetics and toxicity of these drugs have been studied [102,103,[113], [114], [115], [116], [117], [118], [119]]. Based on extensive experimental and clinical trials, the possibility of using autologous erythrocyte ghosts containing an antibiotic and cytokine to improve the results of surgical infection treatment has been proven. Analysis of the dynamics of wound healing and clinical and cytological data revealed a significant acceleration of the healing of purulent wounds with the use of pharmacocytes in contrast to traditional treatment. Studies have demonstrated the possibility of achieving a consistently high concentration of an antibiotic in blood serum and wound areas for a long time upon treatment with pharmacocytes containing a single dose of a drug, in contrast to traditional intravenous administration or local saturation of tissues with the same antibiotic.

The clinical use of erythrocyte carriers for the delivery of therapeutic agents discussed in this article is shown in Table 1.

The article "Drug-loaded erythrocytes: Modern approaches for advanced drug delivery for clinical use" was published in 2023. Journal: Heliyon.

**Table 1:** RBC-encapsulated drugs and clinical applications discussed in this article for targeted delivery.

RBC-incorporated drug	Proposed application	Clinical status	References
Dexamethasone 21-phosphate	Treatment of patients with ulcerative colitis, chronic obstructive pulmonary disorder (COPD), cystic fibrosis, Crohn's disease and ataxia-telangiectasia.	Phase I/II clinical trials.	[32,33,34, 35,36].
Adenosine deaminase (ADA)	Enzyme replacement therapy in patients with adult-type ADA deficiency.	Tested in humans.	[71]
Thymidine phosphorylase (TP)	Treatment of patients affected with mitochondrial neurogastrointestinal encephalopathy for enzyme replacement therapy.	Multi-Centre, Multiple Dose, Open Label Trial. Phase I/II.	[72,80]
l-Asparaginase encapsulated within erythrocytes (GRASPA®)	Acute lymphoblastic leukemia in children and adults.	GRASPALL 2005-01 randomized trial. Phase 2 study.	[40,81]
l-Asparaginase	Pancreatic cancer.	A phase I clinical study.	[79]
Antibiotics (kanamycin and gentamicin, ceftriaxone), hepatoprotectors, cytokines.	Treatment of cholecystitis, peritonitis, purulent wounds (anal abscesses) and septic conditions.	Tested in humans.	[42,43,44, 54,55,56].

## 7 The engineering and technological approaches used in the encapsulation of erythrocytes

Scientific organizations and pharmaceutical companies strive to develop technological solutions for the production of cellular transport systems for targeted drug delivery. The industrial production of cellular transport systems relies on centralized or stationary automated devices, facilitating encapsulation procedures for therapeutic drugs. However, it's crucial to acknowledge the significant hurdles in clinical translation, notably the challenges associated with standardization for large-scale production and the regulatory approval processes. Key issues affecting successful industrialization include production scalability, process validation, and quality control of the produced therapeutic agents. The article [60] discusses both the advantages and disadvantages of various production processes, shedding light on critical success factors in clinical advancements. Despite the legal and regulatory challenges faced in the clinical development of erythrocyte carriers, the industrial sector is making rapid progress in this direction. Several companies have started the development of drug-loaded RBCs using specialized equipment.

Hypo-osmotic drug encapsulation techniques are more suitable procedures for the development of personalized and automated equipment for RBC encapsulation than other RBC loading techniques. As determined from a literature review and patent search, the technological approaches used in the encapsulation of erythrocytes have been revealed and will be discussed further. The authors [120,121] succeeded in using erythrocytes as drug delivery vehicles for magnetic resonance imaging (MRI). Erythrocytes treated with hypotonic dialysis stably absorbed superparamagnetic iron oxide nanoparticles and were used as a contrast agent in MRI. The encapsulation of superparamagnetic nanoparticles in erythrocytes has led to the creation of new biomimetic structures that, when used in vivo, prevent rapid sequestration and accumulation in undesirable areas (WO 2008/003524) [120,121].

The article "Drug-loaded erythrocytes: Modern approaches for advanced drug delivery for clinical use" was published in 2023. Journal: Heliyon.

Indocyanine green (ICG) was encapsulated in human erythrocytes by hypotonic dialysis, isotonic sealing and resealing of the membrane. These steps were carried out using various sterile containers included in the kit. Some containers were disposable centrifuge tubes. The ability of erythrocytes to be preloaded with various substances, such as fluorescent dyes, has facilitated medical imaging using these kits, compositions and methods (Patent US20110098685 A1) [122]. Similarly, the encapsulation of infrared fluorescent agents in erythrocytes allowed the measurement of vasomotor activity in the vascular retina of human eyes, suggesting a possible correlation with retinal edema. Another variant of targeted delivery applies to situations in which the target vascular area is optically accessible, for example, eye vessels or vessels of hollow organs, such as the bladder. Red blood cells loaded with appropriate substances can be delivered by an optical instrument, thus allowing precise delivery to the localized affected areas [123,124]. Bahmani B. et al. [125] achieved a significant breakthrough by successfully engineering hybrid nano-scale structures using membranes derived from erythrocytes depleted of hemoglobin. The near-infrared chromophore, indocyanine green, was encapsulated within these constructs. The authors demonstrated the efficacy of these structures as photo-theranostic agents in fluorescence imaging and photothermal destruction of human cells. These nanostructures, mimicking erythrocytes, can be derived from autologous cells, presenting a vast range of potential applications in personalized nanomedicine. Magnani et al. developed a fully automated device named the “Red Cell Loader” for the encapsulation of human hexokinase and dexamethasone 21-phosphate in RBCs in 1998 [126]. This Red Cell Loader is a highly automated apparatus for drug loading that includes a reusable part equipped with mechanical elements: pumps, valves, electronic units, and a control unit. The apparatus also includes a disposable part, which is adapted to contact erythrocytes and consists of a system of tubes, reservoirs, and filters. The device allows loading of the drug into erythrocytes in a completely automated manner. Dexamethasone sodium phosphate has been encapsulated in human erythrocytes and has been used in the treatment of cystic fibrosis, Crohn's disease, ulcerative colitis, ataxia-telangiectasia, and COPD [[81], [82], [83], [84], [85]]. The results obtained allowed the EMA to recognize dexamethasone sodium phosphate for encapsulation in human erythrocytes as an orphan drug. To date, this device has been improved, and the production of the Red Cell Loader has been established by the company “EryDel” in Italy [127].

The article "Drug-loaded erythrocytes: Modern approaches for advanced drug delivery for clinical use" was published in 2023. Journal: Heliyon.

Bax et al. successfully used the hypotonic dialysis procedure in clinical practice for 17 years in the treatment of patients suffering from adenosine deaminase (ADA) deficiency. Patients were treated at 2- to 3-week intervals with ADA-loaded autologous erythrocytes prepared in dialysis bags. The effectiveness of this treatment has been improved due to the protection of the erythrocyte-encapsulated enzyme from reactions of the anti-ADA neutralizing antibody [128]. The same process of hypo-osmotic dialysis was used to encapsulate thymidine phosphorylase (TP) into erythrocytes, and therapeutic benefits were observed in patients with mitochondrial neurogastrointestinal encephalomyopathy [129].

Both ADA-RBC and TP-RBC preparation processes were applied in accordance with the rules of good manufacturing practice (GMP) in a pharmaceutical environment. However, to achieve industrial production, this loading process using dialysis packages needs to be optimized in terms of storage time, automation and large-scale feasibility.

In subsequent studies, the authors replaced the dialysis bag with a dialysis cartridge consisting of several hollow fibers, which constituted a hemodialyzer, providing much more convenient processing of large volumes of blood. The entrance of drugs into erythrocytes was carried out by contact of a cell suspension with a hypotonic buffer solution flowing in the opposite direction in a hemodialyzer [130,131].

Even earlier, in 1982, Ropars et al. developed the continuous-flow dialysis method for the encapsulation of drugs into RBCs using standard hemodialysis equipment [132]. Then, Ropars et al. patented the automated process of loading drugs into erythrocytes using encapsulation of inositol hexaphosphate (IHP), Patent EP 0101341 [132,133]. Despite the fact that the device guarantees the production of sterile suspensions of erythrocytes without pyrogens, this method has not been tested in clinical practice.

In 2006, Godfrin optimized this automated RBC loading process and developed a device called ERYcaps® for industrial applications (patented technology of ERYTECH Pharma, Lyon, France), Patent WO 2006016247. 2006 Feb. 16 [134]. ERYcaps® allows loading of erythrocytes with a drug in accordance with GMP. In this method, the entire automated drug encapsulation process takes approximately 3 h, and it is possible to load 250–350 ml of erythrocytes. This strategy can be successfully used to increase the half-life of active macromolecules in blood circulation in accordance with the half-life of drug-loaded erythrocytes. Multiple studies have been conducted by Godfrin et al. using this technology for the encapsulation of erythrocytes for enzyme replacement therapy and as enzyme bioreactors in cancer treatment [[134], [135], [136], [137], [138]].

The article "Drug-loaded erythrocytes: Modern approaches for advanced drug delivery for clinical use" was published in 2023. Journal: Heliyon.

A phase I clinical study using l-asparaginase-loaded RBCs in the treatment of pancreatic cancer patients, a phase 2 study of l-asparaginase encapsulated in erythrocytes in patients with acute lymphoblastic leukemia and a multicenter trial of erythrocyte-encapsulated thymidine phosphorylase for the treatment of patients with encephalomyopathy have been conducted.

Based on the method of hypoosmotic dialysis, the authors [139] created a small-volume dialyzer for loading RBCs with enzymes that digest ammonium, which reduces the concentration of ammonium in the blood.

The introduction of targeted drug delivery technology based on pharmacocytes into clinical practice makes it possible to increase the effectiveness of antibacterial treatment of severe cases of surgical infection [93,101,[110], [111], [112]]. Targeted delivery of antibiotics results in the greatest anti-inflammatory effect on the purulent-inflammatory region, reducing overall toxicity due to the selective distribution of drugs in the body.

However, the process of preparing pharmacocytes is laborious since it is performed manually and takes 2.5–3 h. The process of drug loading requires strict compliance with sterile conditions and standardization of technology for the widespread introduction of the innovative treatment method into clinical practice.

Based on the experience gained in using autologous erythrocytes as drug carriers, the authors [[110], [111], [112]] considered that the process of preparing pharmacocytes by hypo-osmotic hemolysis requires optimization by automation of the technology. Automated devices could allow the widespread production of RBC-encapsulated therapeutic drugs for clinical needs.

Automation of the pharmacocyte preparation process would allow us to maintain sterile conditions and standardize loading technologies, as well as facilitate labor-intensive manual work and save staff working time.

The article "Drug-loaded erythrocytes: Modern approaches for advanced drug delivery for clinical use" was published in 2023. Journal: Heliyon.

The authors [[110], [111], [112]] intend to automate the hypo-osmotic hemolysis method used to obtain transport systems for targeted drug delivery based on autologous erythrocytes, which has been performed only manually to date.

The authors [110,112] have started to develop a prototype of an automated software-controlled device with a disposable sterile set of consumables for automatic loading of erythrocytes with selected drugs. The device was designed to operate strictly in accordance with the standard procedure for obtaining pharmacocytes by hypo-osmotic hemolysis.

Automation of the technology for obtaining a transport system based on autologous erythrocyte ghosts ensures the optimization of the process of targeted drug delivery in the body and accelerates the widespread introduction of an innovative treatment method into clinical practice, significantly expanding the effectiveness of treatment both in surgery and in all areas of medicine.

## 8 Conclusion and future perspectives

The use of erythrocytes as drug carriers is a fundamental advance in modern bioengineering and can improve the effectiveness of treatments in many areas of medicine. Hypo-osmotic drug encapsulation techniques are the most suitable procedures for the development of personalized and automated equipment compared to other RBC loading techniques. Advances in the development of automated devices suitable for clinical use based on osmotic methods of loading RBCs have been studied. The accuracy and measurability of osmotic methods of loading drugs into erythrocytes have allowed several commercial companies to develop devices suitable for clinical use.

A patent search revealed two promising technologies with proven clinical therapeutic results from the companies EryDel and ERYTECH. The Red Cell Loader device (EryDel, Italy) was designed to load dexamethasone 21-phosphate by a hypotonic preswelling procedure for the treatment of cystic fibrosis, Crohn's disease, ulcerative colitis, COPD, and ataxia-telangiectasia [126,127]. The ERYcaps® device (ERYTECH Pharma, Lyon, France) was designed for loading asparaginase, inositol hexaphosphate, adenosine deaminase and thymidine phosphorylase by a hypotonic dialysis procedure for the treatment of mitochondrial neurogastrointestinal encephalomyopathy and adenosine deaminase deficiency [[134], [135], [136], [137], [138]]. Glassman PM et al. [13] emphasized that significant drug delivery applications involving RBCs that have advanced to the clinical stage utilize cargo encapsulation within RBCs. It's important to highlight that two promising automated devices with proven clinical therapeutic results and produced by companies EryDel and ERYTECH, also rely on hypo-osmotic loading methods by encapsulating drugs into RBCs.

The article "Drug-loaded erythrocytes: Modern approaches for advanced drug delivery for clinical use" was published in 2023. Journal: Heliyon.

Based on the experience gained in using autologous erythrocytes as drug carriers, the authors [[110], [111], [112]] considered that the process of preparing pharmacocytes by hypo-osmotic hemolysis requires optimization by automation of the technology. Automated devices could provide the widespread production of RBC-encapsulated therapeutic drugs for clinical needs.

Automation of the pharmacocyte preparation process is expected to allow sterile conditions to be maintained and loading technologies to be standardized, as well as to facilitate labor-intensive manual work and save staff working time.

Automation of the technology for obtaining a transport system based on autologous erythrocyte ghosts ensures the optimization of the process of targeted drug delivery in the body and accelerates the widespread introduction of an innovative treatment method into clinical practice, significantly expanding the effectiveness of treatment both in surgery and in all areas of medicine.

Further development of engineering and technological solutions for the automatic production of drug-loaded RBCs for targeted drug delivery for clinical needs is a priority challenge for the pharmaceutical industry.

## Ethics approval and consent to participate

Not applicable.

## Consent for publication

Not applicable.

## Data availability statement

No.

No data was used for the research described in the article.

## Funding

This research is funded by the Science Committee of the Ministry of Science and Higher Education of the Republic of Kazakhstan Grant №AP09258926; №AP19676272and by 10.13039/501100012632Nazarbayev University under Collaborative Research Program Grant № 211123CRP1614, A.G."

## CRediT authorship contribution statement

**Kulzhan Berikkhanova:** Writing – review & editing, Validation, Supervision, Methodology, Investigation, Funding acquisition, Data curation, Conceptualization. **Erlan Taigulov:** Writing – review & editing, Validation, Methodology, Investigation, Data curation, Conceptualization. **Zhanybek Bokebaev:** Writing – original draft, Visualization, Validation, Investigation, Data curation. **Aidar Kusainov:** Writing – original draft, Methodology, Investigation, Data curation. **Gulyash Tanysheva:** Writing – original draft, Visualization, Methodology, Investigation, Data curation, Conceptualization. **Azamat Yedrissov:** Writing – review & editing, Validation, Methodology, Investigation, Data curation, Conceptualization. **German Seredin:** Writing – review & editing, Visualization, Validation, Methodology, Investigation, Data curation, Conceptualization. **Tolkyn Baltabayeva:** Writing – review & editing, Methodology, Investigation, Data curation, Conceptualization. **Zhaxybay Zhumadilov:** Writing – review & editing, Supervision, Methodology, Conceptualization.

The article "Drug-loaded erythrocytes: Modern approaches for advanced drug delivery for clinical use" was published in 2023. Journal: Heliyon.

## Declaration of competing interest

The authors declare that they have no known competing financial interests or personal relationships that could have appeared to influence the work reported in this paper.

## List of abbreviations

RBCs: red blood cells
ATP: adenosine triphosphate
RCNPs: RBC membrane-camouflaged nanoparticles
RCNPs: red blood cell-derived extracellular vesicles
hTM: human thrombomodulin
suPAR: soluble urokinase plasminogen activator receptor
PAI-1: plasminogen activator inhibitor-1
tPA: tissue-type plasminogen activator
AuNPs: amphiphilic gold nanoparticles
RH: RBC-hitchhiking
NCs: nanocarriers
DTRH: Dual Targeted RBC Hitchhiking
PK: pharmacokinetics
ADME: absorption, distribution, metabolism, elimination
PEGylation: coating nanoparticles with polymers polyethylene glycol
GPA: glycophorin A
PS: phosphatidylserine
ROS: reactive oxygen species
NIR: near-infrared
PB: Prussian blue
Ce6: Chlorin e6
RBCM: Red blood cell membranes
RBCEVs: Extracellular vesicles
Abs: antibodies
CPZ: chlorpromazine
PMCA: plasma membrane Ca2+-ATPase
SDS-PAGE: sodium dodecyl sulfate-polyacrylamide gel electrophoresis
DAF: decay accelerating factor
DMSO: dimethyl sulfoxide
DNA: deoxyribonucleic acid
RES: reticuloendothelial system
EMA: European Medicines Agency
COPD: chronic obstructive pulmonary disorder
Dexa 21-P: derivative corticosteroid dexamethasone 21-phosphate
MRI: magnetic resonance imaging
ICG: indocyanine green
ADA: adenosine deaminase
TP: thymidine phosphorylase
GMP: good manufacturing practice
IHP: inositol hexaphosphate
